The article "Manipulative Reduction for Abnormal Uterine Inclination in Vaginal Delivery" was published in 2022. Journal: Comput Math Methods Med.

# Manipulative Reduction for Abnormal Uterine Inclination in Vaginal Delivery

**DOI:** 10.1155/2022/4765447

**Published:** 2022-01-30

**Authors:** Jia Chen, Yujuan Yuan, Yadong Wang

**Affiliations:** ^1^Department of Obstetrics and Gynecology, Chongqing University Central Hospital (Chongqing Emergency Medical Center), Chongqing 400014, China; ^2^Department of Galactophore, Chongqing Traditional Chinese Medicine Hospital, Chongqing 400021, China

## Abstract

**Objective:**

To investigate the manipulative reduction in abnormal uterine inclination in vaginal delivery.

**Methods:**

With the independently developed uterine inclination surveyor, 40 primiparas with abnormal uterine inclination were randomly divided into two groups: treatment group (Group A, 20 cases) and control group (Group B, 20 cases). The general condition of the primipara, the labor stages, the changes in uterine inclination after treatment, postpartum hemorrhage at 2 hours, and the general condition of fetuses were observed to study the therapeutic value of manual reduction in abnormal uterine inclination.

**Result:**

In the control group, one uterine inclination was not corrected with the change in labor process, and the pregnancy was terminated due to stagnation of the active phase. In the first stage of labor, the time spent in the treatment group (393.4 ± 31.3 mins) was significantly lower than that in the control group (440.7 ± 34.9 mins) (*P* = 0.001). Compared with the control group (49.8 ± 6.5 mins), the treatment group (42.6 ± 7.2 mins) also exhibited a significantly shortened second stage of labor (*P* = 0.02). Sixteen cases (16/20) in the treatment group returned to normal after manual reduction, and 9 cases (9/20) in the control group returned to normal with the progression of natural labor. Manual reduction could be used as an option to treat abnormal uterine inclination (*P* = 0.01). There was no significant difference in the third stage of labor (*P* = 0.2), 2-hour postpartum hemorrhage (*P* = 0.35), Apgar score (*P* = 0.64), or body weight (*P* = 0.76) between the two groups.

**Conclusion:**

Manual reduction in the treatment of abnormal uterine inclination has obvious effects, shortens the birth process, and is safe for the fetus.

## 1. Introduction

Dystocia is a broad term, statistically defined as the rate of cervical dilatation which is lower than 95% of normal delivery. The treatment of dystocia is limited to increasing oxytocin. If cervical dilatation continues to be insufficient, cesarean section will be performed. Nonetheless, about 12% of women do not respond adequately to increased oxytocin, indicating changes in the underlying pathophysiology of dystocia [1]. Monitoring uterine activity is a common component of both the diagnosis and management of labor dystocia. Active management of labor dystocia typically includes calculating adequacy of uterine contractions using Montevideo units (MVUs) measured via an intrauterine pressure catheter [2]. Studies have found that the inclination of the pelvis and uterus in the birth canal is also an influential factor in dystocia [3]. Uterine inclination is an important factor for birth canals and fetuses in vaginal delivery [4]. Fetal axis inclination is the angle between the longitudinal axis of the pregnant woman and the fetus without fetal movement and contraction. Uterine inclination (Figure 1) is the angle between the longitudinal axis of the pregnant woman and the uterus without fetal movement and contraction [3]. There was no significant difference between the uterine inclination and the fetal axis inclination; in other words, the uterine inclination was the same as the fetal axis inclination. Related studies suggest that abnormal uterine inclination may lead to prolonged labor or even stagnation and may require a cesarean section to terminate the pregnancy. Till now, no data were found on the association between restoration of the uterine axis and vaginal delivery. In this study, abnormal uterine inclination was treated by manual restoration of the uterine axis, and its effect was explored.

## 2. Materials and Methods

### 2.1. Case Selection and Groups

40 cases of primiparous women were selected at Chongqing Municipal Emergency Medical Center/Chongqing Municipal Fourth People's Hospital from May 2018 to November 2019: women aged 20 to 40 years, 155 to 180 cm in height, 50 to 80 kg in weight, no hypertension and diabetes, single fetus, full-term (greater than or equal to 37 weeks, less than 41 weeks), voluntary enrollment, in line with the requirements of labor vaginal, uterine inclination (greater than 3°, less than or equal to 17°). They were randomly divided into a treatment group (group A) and a control group (group B). 20 women were included in each group.

### 2.2. Measurement of Uterine Inclination

With a uterine inclination measuring instrument (National patent number: 201720408894.7, Figures 2 and 3), which has been independently and successfully researched and developed [5], the uterine inclination is measured when the uterine opening is larger than 3 cm, without uterine contraction. Eligible pregnant women (uterine inclination greater than 3° and less than or equal to 17°) were randomly divided into a treatment group and a control group.

### 2.3. Resetting of the Fetal Axis by Hand

To meet the conditions of uterine inclination, a professionally trained midwife performs a manual reduction before the contractions start. The professionally trained designated midwife stands on the affected side. If midwives stand on the left side, their right hand is placed on the uterine floor to fix it, and their left hand is placed on the right side of the uterus to slowly increase the force until the uterine inclination is almost normal, stopping when uterine contractions occur. When standing on the right, the opposite placements are applicable. The intervention can be repeated 4 to 6 times, and the recovery of the uterine inclination is evaluated every 2 times. The intervention is stopped when the uterine inclination is less than 3°. The above operations are performed on Group A but not Group B.

### 2.4. Observation Data

The data were acquired with the uterine inclination-measuring instrument, including 3 cm and 1 hour later, as well as the changes after manual intervention every 2 times. Information on general condition of the primipara, labor stages, changes in uterine inclination after treatment, postpartum hemorrhage at 2 hours, the general condition of the fetus, and Apgar scores was collected.

### 2.5. Statistical Analysis

Statistical analysis was carried out with GraphPad Prism 6.0 (GraphPad Software, La Jolla, CA, USA). The data are shown as the mean ± SD. Categorical variables were examined for association using Pearson's *χ*^2^ and Student's 2-sample *t*-test. Differences were considered significant at *P* < 0.05.

### 2.6. Institutional Review Board Approval

All patients involved in this study signed informed consent. Approval from the Institutional Review Board of our hospital was obtained for this study.

## 3. Results

### 3.1. General Situation

Eligible pregnant women had an average age of 29 years, a height of 1.62 m, a birth weight of 67 kg, and a delivery time of 39 weeks. The uterine inclination was 9° on average in both groups. Age (*P* = 0.85), height (*P* = 0.56), weight (*P* = 0.41), gestational week (*P* = 0.52), and uterine inclination (*P* = 0.51) were compared between the two groups, without a significant difference (Table 1). The influence of uterine inclination receptor weight and height was confirmed, and this study found no obvious correlation between the two groups. This experiment did not detect any evidence that there was no significant difference between the treatment and control groups in the basic situation.

### 3.2. The Postpartum Performance of the Treatment and Control Groups

In the control group without manual intervention, there was one pregnant woman whose uterine inclination was 10°; the active stage of labor stagnated, and the pregnancy was terminated by cesarean section. In the first stage of labor, the time in Group A was 393.4 ± 31.3 mins, while the time in Group B was 440.7 ± 34.9 mins. The difference between the two groups was significant (*P* = 0.001). The average time of the second labor stage in the 20 cases in the treatment group was 42.6 ± 7.2 mins, while the average time in the 19 cases in the control group was 49.8 ± 6.5 mins. The *t*-test was performed on the two groups, and the results showed a statistically significant difference (*P* = 0.02). By manual reduction, the second stage of labor was significantly shortened. Correcting abnormal uterine inclination in time may avoid difficult labor. In the third stage of labor, the average time (9.9 mins) of the treatment group was shorter than that of the control group (11.0 mins); however, there was no significant difference between the two groups (*P* = 0.2). In the results of this study, contrary to our prediction, there was no significant difference between the two groups (*P* = 0.35), and manual intervention did not significantly reduce the amount of postpartum hemorrhage (Table 2).

### 3.3. Comparison of Changes in Uterine Inclination before and after Intervention in the Treatment Group

When the cervical opening was larger than 3 cm, the uterine inclination of the treatment group was 9.8 ± 2.6°, while that of the control group was 9.2 ± 3.0°, without a statistically significant difference (*P* = 0.51). When entering the second stage of labor, the uterine inclination was measured again. The uterine inclination was less than 3° in 16 of 20 cases in the treatment group and in 9 of 20 cases in the control group. This study showed that there was a significant difference between the two groups (*P* = 0.01, Figure 4).

### 3.4. Postpartum Fetal Condition

During delivery, the weight of newborns in the treatment group was 3.36 ± 0.23 kg, while that in the control group was 3.34 ± 0.28 kg. There was no significant difference between them (*P* = 0.76). The influence of uterine inclination on the second stage of labor may lead to a lower Apgar score in newborns. However, this study showed that there was no statistically significant difference between the Apgar scores in the treatment group (9.85 ± 0.37) and the control group (9.90 ± 0.31) (*P* = 0.64) (Table 2).

## 4. Discussion

Dystocia is the most common cause of cesarean delivery in obstetrics, but how it develops during delivery remains elusive. Uterine activity monitoring has great potential to advance our understanding of dystocia. Assessing the frequency and magnitude of contractions is a common component of dystocia management. Management of dystocia has been identified as an opportunity for reducing the unnecessary cesarean rate and the associated risks to women and their infants [6]. With rich practical care experience and useful prediction data, the discussion of the contextualized discussions of shared decision-making in what is most meaningful to women is more specific and accurate, and the decision errors caused by the differences in dystocia methods are minimized [7]. In addition, many high-income countries (HICs) and more low- and middle-income countries (LMICs) are undergoing “obstetric transition” [8, 9]. This is a concept regarding the long-term trend of declining fertility and maternal mortality. Some researchers believe that this transition is also the result of the aging obstetric population and a movement from the natural history of pregnancy to the medicalization of maternity care. To reduce the rate of cesarean section and the fear of pregnant women regarding childbirth, the monitoring and regulation of natural childbirth should be more clinically inclined [10]. This study is aimed at making the birth process smoother by detecting a new index (uterine inclination), detecting the process of natural delivery, and promptly intervening in abnormal patients.

Dystocia is common and a high-risk problem in obstetrics. There are countless variables that can cause dystocia. Demographic factors, such as maternal age, and clinical factors, such as body mass index, fetal position, fetal age, estimated fetal weight, use of epidural analgesics, and induction of labor, may lead to dystocia and subsequent medical or surgical intervention. Increasing maternal age and obesity are two increasingly common factors among women of childbearing age. They are speculated to have an impact on uterine contractility, thus increasing the risk of dystocia [11, 12]. In addition to the accident of pelvic stenosis in the birth canal, Ling Luoda found that the size of the pelvic inclination is also one of the factors of dystocia. The pelvic inclination measuring instrument was invented using the human body structure [11, 12]. Sun Jiangchuan found that uterine inclination also has a certain effect on vaginal delivery and even causes dystocia without timely treatment. The purpose of this study was to explore whether the abnormal inclination of the uterus can effectively improve and change the birth process through manual reduction to provide new evidence for dystocia and further reduce the cesarean section rate [13].

According to the requirements, 40 cases were randomly divided into a treatment group and a control group. There was no significant difference in age, height, weight, gestational age, or degree of uterine inclination between the two groups. The abnormality of the fetal position can be corrected by manual intervention. For instance, fetal occiput posterior (OP) positions account for 15 to 20% of cephalic presentations and are associated with poorer maternal and neonatal outcomes than occiput anterior (OA) positions [14–17].

In the process of delivery, the parturient corrected the position of the fetus by adjusting the posture and medical treatment to make the delivery smooth. The longitudinal lie is classified as a normal mode, and the transverse lie is mostly reported in the second fetal mode of twins. In addition to the controversy regarding the transverse lie of twins, the majority of opinions on the transverse involve caesarean section [18]. However, for the abnormal mode of labor between the longitudinal lie and the transverse lie, called abnormal uterine inclination in this study, manual reduction is recommended clinically. In this study, manual reduction in the treatment group shortened the first and second stages of labor, but the effect on the third stage of labor was not obvious. For both the pregnant woman and the midwife, the second stage of labor is the most stressful part of the delivery process. Management of the second stage of labor is the primary responsibility of the midwife. For some pregnant women, the second stage of labor may be beneficial in promoting the best maternal and neonatal outcomes [6]. Through intervention of the labor process, this study arrived at similar results as previous authors. In the control group, for one woman, the uterine inclination did not change with the process of delivery, as it was measured at 10° during both tests. Her pregnancy was terminated by cesarean section due to stagnation of the active phase. This phenomenon may be due to abnormal uterine inclination, which can lead to stagnation of the active stage of labor. However, there is a lack of additional indicators to support this hypothesis, which requires further study. Unexpectedly, there were no significant differences in postpartum hemorrhage at 2 hours, Apgar score, or fetal weight. Although it cannot be concluded that abnormal uterine inclination affects the outcome of delivery, it can explain the safety of manual reduction in vaginal delivery.

Taken together, we explored the association of restoration of the uterine axis with vaginal delivery and found manual restoration of the uterine axis could rescue abnormal uterine inclination. In such case, manual reduction in the treatment of abnormal uterine inclination has obvious effects, shortens the birth process, and is safe for the fetus. This study can further improve the role of drugs such as oxytocin in abnormal uterine inclination and the safety of vaginal delivery. In the future, whenever possible, women with obesity and of advanced maternal age should be included in the study, and other covariates should be considered in the analysis to evaluate the measurement of uterine activity and its relationship with outcome variables, including dystocia and cesarean section, so as to understand how these variables affect the pathophysiology of dystocia.

## Figures and Tables

**Figure 1:** Projection of the human body at the uterine inclination. Point O is the upper edge of the pubic symphysis, point A is the point below the anterior midline xiphoid, and point B is the actual uterine floor position. Line OA is the midline of the human body, line OB is the longitudinal axis of the uterus, and the angle *α* is the uterine inclination as defined in this study.

**Figure 2:** Uterine inclination measuring instrument. A: side view; B: top view. Notes: the uterine inclination measuring instrument consists of the following parts: (1) fixed base, (2) fixed support, (3) transverse support rod, (4) measuring plate, (5) measuring structure, (51) pointer part, (52) projection part, (6) housing, (7) cantilever line, (8) suspended hammer, (81) suspended hammer, and (8) button.

**Figure 3:** Uterine inclination measuring instrument (top view).

**Figure 4:** Comparison of the curative effect between Group A and Group B (*n* = 40). ∗ indicates a statistically significant difference (*P* < 0.05).

**Table 1:** Individual characteristics according to occurrence in Group A and Group B during labor (*N* = 40, mean ± SD).

Characteristics	Group A	Group B	*P* value^a^
General information			
Age (years)	28.45 ± 4.25	28.75 ± 5.75	0.85
Height (cm)	158.0 ± 4.21	157.2 ± 4.44	0.56
Weight (kg)	66.75 ± 9.40	69.08 ± 8.38	0.41
Prenatal fetal information			
Gestational age (weeks)	39.64 ± 0.74	39.48 ± 0.75	0.52
UI (degree)	9.8 ± 2.6	9.2 ± 3.0	0.51

^a^Using Pearson's *χ*^2^ test and Student's 2-sample *t*-test as appropriate.

**Table 2:** Changes in pregnant women and fetuses in the course of childbirth in Group A (*n* = 20, mean ± SD) and Group B (*n* = 20, mean ± SD).

Characteristics	Group A	Group B	*P* value^a^
Labor process			
The first stage (min)^b^	393.4 ± 31.3	440.7 ± 34.9	0.001
The second stage (min)^b^	42.6 ± 7.2	49.8 ± 6.5	0.02
The third stage (min)^b^	9.9 ± 2.0	11.0 ± 3.1	0.20
Postpartum hemorrhage			
Postpartum hemorrhage at 2 hours (ml)	76.4 ± 20.1	80.1 ± 16.8	0.35
The fetus			
Neonatal weight (kg)	3.36 ± 0.23	3.34 ± 0.28	0.76
Apgar score	9.85 ± 0.37	9.90 ± 0.31	0.64

^a^Using Pearson's *χ*^2^ test and Student's 2-sample *t*-test as appropriate. ^b^Using *n* = 19 in group B; one sample was terminated by cesarean section on account of active phase arrest.

## Data Availability

The authors confirm that the data supporting the findings of this study are available within the article.
